# K-Means Clustering Algorithm–Based Functional Magnetic Resonance for Evaluation of Regular Hemodialysis on Brain Function of Patients with End-Stage Renal Disease

**DOI:** 10.1155/2022/1181030

**Published:** 2022-06-21

**Authors:** Yan Cheng, Yan Yu

**Affiliations:** ^1^Department of Nephrology, The Third People's Hospital of Zhengzhou, Zhengzhou, 453000 Henan, China; ^2^Department of Nephrology, Affiliated Hospital of Nantong University, Nantong, 226001 Jiangsu, China

## Abstract

This research was to evaluate the effects of regular hemodialysis (HD) on the brain function of patients with end-stage renal disease (ESRD). Resting-state functional magnetic resonance imaging (rs-fMRI) based on improved k-means clustering algorithm (k-means) was proposed to scan the brains of 30 regular dialysis patients with end-stage renal disease (ESRD) (experimental group) and 30 normal volunteers (control group). The proposed algorithm was compared with the traditional k-means algorithm and mean shift algorithm and applied to the magnetic resonance scan of patients with ESRD on long-term regular HD. The results showed that the neuropsychological cognitive function (NSCF) evaluation result of the test group was much better than that of the control group, and the difference was statistically obvious (*P* < 0.05). The results of blood biochemistry, Digit Symbol Substitution Test (DSST), and Montreal Cognitive Assessment Scale (MoCA) in the test group showed no statistical difference compared with those in the control group. The running time of the improved k-means algorithm was dramatically shorter than that of traditional k-means algorithm, showing statistical difference (*P* < 0.05). Comparison among the improved and traditional k-means algorithm and mean shift algorithm suggested that the improved k-means algorithm showed a lower error rate for image segmentation, and the differences were statistically remarkable (*P* < 0.05). In conclusion, the improved k-means algorithm showed better time efficiency and the lowest error rate in processing rs-fMRI images than the traditional k-means algorithm and mean shift algorithm, and the effects of regular HD on the brains of patients with ESRD were evaluated effectively.

## 1. Introduction

End-stage renal disease (ESRD) refers to the endogenous creatinine clearance rate of the patient is less than 15 mL/(min 1.73 m^2^) for continuous 3 months or more [1]. The morbidity and mortality of ESRD have attracted the attention of relevant scholars around the world [2, 3]. Studies have shown that the incidence of cognitive impairment in the complications of ESRD patients accounts for about 15% ~32% of all patients, but the pathological mechanism of how to cause brain damage in patients with cognitive dysfunction is currently unclear [4]. For most ESRD patients, HD is a common treatment to prolong the survival time of patients, but HD is not only a traumatic treatment but also causes psychological discomfort to patients. According to related reports, the risk of cognitive dysfunction in patients receiving HD treatment is as high as 60%, and most patients may have cognitive dysfunction in the early stage, such as coordination movement disorder, memory decline, executive disorder, and control ability disorder [5]. In the later stages of the disease, as the frequency of HD treatment continues to increase, patients may experience severe neurological damage, such as brain atrophy and cerebral infarction [6]. Therefore, how to quickly detect and diagnose the symptoms and signs of the early nervous system of ESRD patients, improve the prognosis of the patients, and reduce the mortality of the disease are the key issues of many scholars.

At present, there are few methods for evaluating the nervous system damage of ESRD patients and analyzing the cognitive dysfunction of patients receiving HD treatment, and most of the evaluation and analysis methods are cumbersome and the judgment results are inaccurate [7]. Some scholars are inspired by the application of magnetic resonance imaging (MRI) to the brain nervous system, suggesting that ESRD patients can use MRI for head examination before and after HD treatment, and then compare the characteristic changes of head MRI before and after treatment [8, 9]. Although MRI head examination is more sensitive to some organic brain lesions, it has deficiencies in some minor lesions, such as microvascular lesions [10, 11]. The emergence of resting-state functional MRI (rs-fMRI) has been widely used in neurology. Compared with MRI, rs-fMRI has high temporal and spatial resolution, and its principle is to use the brain blood oxygen level-dependent effect. Under the stimulation of external factors, the hemoglobin concentration in different brain regions will change, which will cause the magnetic susceptibility around the corresponding part to also change, resulting in a change in the blood oxygen level dependent (BOLD) signal; and rs-fMRI indirectly reflects the brain activity under external stimuli by measuring the change of BOLD signal [12–14]. rs-fMRI cannot be restricted by test requirements and command tasks, its operation is simple, and reproducibility is high, so it can provide a reliable basis for the early and late development of ESRD patients [15].

Although rs-fMRI can bring convenience to the clinical diagnosis and treatment of ESRD patients with neurological disorders, its image segmentation is still affected by the equipment itself and external factors. Regarding how to accurately segment MRI images, some scholars have applied clustering algorithms [16–19]. The k-means clustering (k-means) algorithm is a simple iterative clustering algorithm that uses distance as a similarity indicator to find K classes in a given data set. The center of each class is obtained according to the mean of all the values in the class, and the center of each class is described by the cluster center. The algorithm overly relies on the choice of the initial center, is more sensitive to skew distribution, and easily loses some tiny clustering data [20–23].

To sum up, the trend of k-means for data image processing is increasing, but the algorithm is less researched in the module of rs-fMRI to diagnose the impact of regular HD on the brain function of ESRD patients. Moreover, due to the limitations of this algorithm, there are many defects in clinical application. As a result, the k-means algorithm was improved and applied in the diagnosis of ESRD patients with rs-fMRI in this research. In addition, the mean shift algorithm, the original k-means algorithm, and the improved k-means algorithm were compared to prove the superiority of the proposed algorithm. What's more, effects of regular HD on the cognitive neurological function of ESRD patients were analyzed by dividing the subjects into a test group and a control group and scanning the brains of all subjects with rs-fMRI.

## 2. Materials and Methods

### 2.1. Research Objects

Experimental group: a total of 30 ESRD patients who received regular HD treatment at the hospital from June 2018 to June 2020 were screened, and they all met the requirements of the test, including 13 females and 17 males. Control group: 30 volunteers from the hospital were selected during the same period. After physical examination, 30 volunteers were healthy, including 14 males and 16 females. This research had been approved by the ethics committee of the hospital. All participants signed the written informed consent forms and volunteered to participate in this research.

### 2.2. Inclusion and Exclusion Criteria

The inclusion criteria for patients in the test group were given as follows: patients with complete clinical data related to the trial; patients with ESRD, and the diagnostic criteria of which met the internationally recognized chronic kidney disease guidelines formulated by the American Kidney Foundation; patients aged 40~60 years old; patients with education years of more than 6 years; patients who were right-handed; and patients who signed the informed consent forms. The exclusion criteria were given as follows: patients with complicated major diseases, such as severe myocardial infarction, cerebral infarction, and heart disease; patients with severe mental disorders that cannot cooperate with the trial; patients with pacemakers who were not suitable for MRI; patients with left-handedness; and patients who had not signed the informed consents.

The inclusion criteria for subjects in the control group were described as follows: those whose basic clinical data met the screening requirements of the trial; those who did not suffer from major diseases; those who were right-handed volunteers; and those who had signed the informed consents, while the exclusion criteria were defined as those who were unwilling to cooperate with the test; those who had major diseases; those who were severely addicted to tobacco and alcohol; those who were not suitable for MRI; and those who had not signed the informed consents.

### 2.3. Neuropsychological Test

Three hours before receiving the rs-fMRI scan of the brain, subjects in both groups received the Digital Symbol Substitution Test (DSST) and Montreal Cognitive Assessment (MoCA). The test time and environment for the two groups of subjects should be kept as same as possible, and the researchers who assisted in the test can strictly follow the specific operations and scoring instructions of the two scales. The main content of the DSST test was visual memory ability, thinking activity, and attention. The test contents of the MoCA scale included attention and concentration, executive ability, memory, language, visual structure branch ability, abstract thinking, calculation ability, and orientation ability.

### 2.4. K-Means Algorithm

The principle of the initial k-means algorithm is to classify data sets into different categories through an iterative process, so as to optimize the clustering ability. This is an iterative process that keeps the cluster center moving. It moves the cluster center to the average position of the cluster including pixels and then resegments the members within the cluster.  Figure 1 is a demonstration of the clustering process using the k-means algorithm.

Although the k-means algorithm can classify data sets through continuous iteration, it cannot determine its own K value, so the initial cluster center must be determined before the surgery. The human brain is composed of many tissues and blood vessels. When MRI scans the brain, the initial clustering can be bone, soft tissue, fat, regional background, etc. It can get the image as shown in Figure 2.

The basic idea of the k-means algorithm is to divide the data into K categories on the basis of minimizing the error function. The processing process of the algorithm was described as follows. Firstly, the initial cluster center and the number of K initial clusters were defined, and then each data in the data set was assigned to the nearest cluster center according to the proposed standard. If the data set *Y* = {*x*_1_, *x*, *x*_3_⋯⋯*x*_*i*_ ⋯ *x*_*n*_} was divided into K categories, the cluster center was *M* = {*c*_1_, *c*_2_⋯, *c*_*N*_⋯, *c*_*K*_}. The data *d*_iN_(*x*_*i*_, *c*_*N*_) was to represent the distance between *x*_*i*_ and its corresponding cluster center *c*_*j*_, and the sum of the distances between all data points in the data set and the type of cluster center could be represented by the objective function *H*:

(1) $$\begin{array}{c} H=\underset{h=1}{\overset{K}{\Sigma }}\underset{i,i\epsilon c_{h}}{\Sigma }d_{ih}\left(x_{i},c_{h}\right). \end{array}$$

The smaller the objective function *H*, the more compact the clustering and the better the clustering quality. When the Euclidean distance was selected as the distance between the data *x*_*i*_ and its corresponding center *c*_*h*_*h*, *x*_*i*_^*h*^ was the data sample belonging to cluster *h*, and *n*_*h*_ was the number of samples in cluster *h*:

(2) $$\begin{array}{c} H=\underset{h=1}{\overset{\text{K}}{\Sigma }}H_{n}=\underset{h=1}{\overset{K}{\Sigma }}\left[\underset{i,i\epsilon c_{h}}{\Sigma }{\left\|x_{i}^{h}-c_{h}\right\|}^{2}\right]. \end{array}$$

To minimize the objective function, each cluster center can be expressed as follows:

(3) $$\begin{array}{c} c_{h}=\frac{1}{n_{j}}\underset{i=1}{\overset{n_{h}}{\Sigma }}x_{i}^{h}. \end{array}$$

After the self-defined cluster center k-means algorithm was improved, the algorithm flow is shown in Figure 3:

### 2.5. MRI Examination

The rs-fMRI images of all the research subjects were acquired with 3.0T MRI scanner, and the head coil was a 12-channel phased array. The scanning process was strictly controlled and operated by a member and sequence. The ordinary MRI detection was performed on the brain of all subjects. The scan sequence included axial T2-weighted imaging, fluid-attеnuatеd invеrsiоn rесоvеry (FLAIR) imaging, diffusion-weighted imaging (DWI), and high-definition sagittal T1-weighted imaging sequence, excluding craniocerebral tumors, cerebral parenchymal hemorrhage, acute and old cerebral infarction, and brain trauma, and other organic diseases. The earplugs were put in the subject's ears before scanning to reduce scanner noise, prevent head movement, and minimize movement artifacts. During the scanning process, the persons were required to close their eyes, breathe calmly, and were in a relaxed state without any thinking or sleep.

Preprocessing is to select statistical parametric mapping (SPM) 12.0 software, REST software package, and data processing assistant for resting-state fMRI (DPARSF) under the matrix laboratory (Matlab) 2012 software platform the software conducts process-style exploration on RS-fMRI data. The experienced brain personnel was arranged to perform manual analysis and evaluation of the scanned images.

### 2.6. Observation Indicators

The relevant clinical data of all subjects were collected. All patients with ESRD underwent blood testing to check various biochemical indicators: serum potassium (K), serum calcium (Ca), serum creatinine (SCr), blood urea nitrogen (BUN), total cholesterol (TC), hemoglobin (Hb), and red blood cell (RBC). All subjects completed neuropsychological cognitive function assessments, including the MoCA scoring scale. All subjects completed rs-fMRI scans, and ESRD patients completed rs-fMRI scans before blood collection.

### 2.7. Statistical Analysis

The SPSS 22.0 software was used to statistically analyze the differences in relevant clinical data, blood biochemistry test results, and neuropsychological test results between the two groups. The normality and homogeneity of variance tests were performed on the measurement data of the two groups of age, education level, neurocognitive scores, and blood biochemical indicators, and the data complying the normal distribution were expressed in the form of mean ± standard deviation, while data not complying the normal distribution were described in the form of median/quartile. When indicators of two groups were compared, two independent sample *t* test (data obey normal distribution and uniform variance), rank sum test (two groups of data do not conform to normal distribution or conform to normal distribution but uneven variance), and chi-square test (compared to gender) were adopted. The two-sample *t*-test was adopted to test the difference in the data components between the two groups, ignoring the covariates such as age, gender, and educational level, and the union of the single-sample *t*-test results was adopted to compare only the DMN components. When *P* < 0.05, the difference was considered to be statistically significant, the Alpha Sim correction was adopted, and cluster size was >49. *P* < 0.05 indicated that the difference was statistically significant.

## 3. Results

### 3.1. Comparison on Running Time of Improved and Traditional K-Means Algorithms

The improved k-means algorithm for customizing the initial center and the traditional k-means algorithm was adopted to process the two 256 × 256 images and two MRI brain scans with a size of 512 × 512 simultaneously. As shown in Figure 4, the improved k-means algorithm was up to 8 seconds faster than the traditional k-means algorithm, and the difference was statistically visible (*P* < 0.05).

### 3.2. Comparison on Segmentation Error Rate among the Traditional and Improved K-Means Algorithm and Mean Shift Algorithm

The mean shift algorithm [24] was introduced and compared with the improved and traditional k-means algorithms in the term of segmentation error rate, and the results are illustrated in Figure 5. It was found that among the three algorithms, the segmentation error rate was the lowest for the improved k-means algorithm proposed in this research, which was 16.3%; the highest segmentation error rate was found in the traditional k-means algorithm (25.33%); and that of the mean shift algorithm was centered at 19.2%. As shown in Figure 5, the differences were statistically significant (*P* < 0.05).

### 3.3. Basic Clinical Data of the Two Groups of Subjects

There were 60 subjects in this research, including 30 ESRD patients in the test group and 30 volunteers in the control group. There were 13 females and 17 males in the test group, and 14 females and 16 males in the control group. The average age of patients in the test group was 52.34 ± 10.23 years old, the average course of disease was 6.63 ± 1.74 years, the average years of education were 10.03 ± 3.27 years, the average height was 16.5 ± 3.08 dm, and the average weight was 62.43 ± 8.64 kg. The average age, years of education, height, and weight of patients in the control group were 49.37 ± 12.13 years old, 10.11 ± 3.46 years, 16.6 ± 4.15 dm, and 63.56 ± 9.08 kg, respectively. As shown in Figure 6, there was no observable difference between the two groups of subjects in age, years of education, height, and weight (*P* > 0.05).

### 3.4. Test on Neuropsychological Cognitive Outcome

The subjects in test group and the control group were tested on the DSST scale and the MoCA scale before the rs-fMRI scan. The test group showed an average of 31.3 points on the DSST scale and an average of 22.43 points on the MoCA scale, while the DSST scale averaged 45.6 points, and the MoCA scale averaged 27.36 points in the control group. As shown in Figure 7, the test results of the DSST scale and MoCA scale were greatly different between the two groups (*P* < 0.05).

### 3.5. Correlation between Psychological Test and Blood Biochemistry Test Results

The correlation between the blood biochemistry results obtained after blood sampling and the DSST scale and MoCA scale was analyzed. It was found that the correlation coefficients between MMAE scale and K, Ca, SCr, BUN, TC, Hb, and RBC were -0.01, -0.25, -0.04, -0.117, 0.22, 0.071, and 0.09, respectively, while the correlation coefficients between MoCA scale and K, Ca, SCr, BUN, TC, Hb, and RBC were -0.22, -0.33, -0.01, -0.112, 0.12, 0.18, and 0.13, respectively. As illustrated in Figure 8, there was no statistically remarkable correlation between the blood biochemistry results and the test results of the DSST scale and the MoCA scale (*P* >0.05).

### 3.6. Analysis on the Difference in Functional Connectivity between Two Groups

Two-sample *t*-test was performed on both the test group and the control group to obtain the functional connectivity difference diagram of the two, as shown in Figure 9. Compared with the control group, the brain area with reduced functional connectivity was located in the precuneus/posterior cingulate gyrus, and the increased brain area was located in the right medial prefrontal cortex in the test group; in addition, the functional connectivity of the different brain areas was statistically significant (*P* < 0.05).

## 4. Discussion

In this research, the basic clinical data of the subjects in different groups were compared, and the results showed that the differences between the two in gender, age, height, and weight were not significant statistically (*P* > 0.05). The results of the DSST scale and MoCA scale of the two groups of subjects were compared, and the results showed that the neuropsychological cognitive test scores of ESRD patients were much lower than those of the control group, showing statistically obvious difference (*P* < 0.05). In addition, the correlation between neuropsychological cognition results and blood biochemistry examination results of ESRD patients was analyzed. The results revealed that the two were not related and the difference was not statistically remarkable (*P* > 0.05). HD treatment is an important therapy to extend the life of ESRD patients, and the filtration of metabolites in patients is still not perfect. The results suggested that the SCr and BUN levels in ESRD patients after HD treatment were relatively high. The previous studies showed that SCr and BUN were related to the damage of the brain function system in patients with ESRD [25, 26]. After discussion, the main reason for the difference between this research and the previous results is that the patients also received HD treatment during the rs-fMRI examination. Oliveira et al. [27] used the low-frequency oscillation amplitude algorithm to research the fMRI of ERSD patients during HD treatment and found the difference between the ESRD patient group and the healthy control group was not obviously connected with SCr and BUN. The reason for this result may be that the SCr and BUN levels of ESRD patients are controlled at relatively stable values during regular HD, and the brain activity of ESRD patients has a certain tolerance to long-term high SCr and bun levels. Sprick et al. [28] showed that ESRD patients undergoing maintenance hemodialysis have multiple cognitive impairments, such as cognitive fluctuations, and the main clinical manifestation is the improvement of executive ability, which may be related to changes in the accumulation of toxic metabolites in ESRD patients during HD [29].

Besides, the comparison on running time showed that regardless of the size of the image, the k-means algorithm based on custom clustering centers was more efficient, which was similar to the results of Krishan et al. [30]. The traditional k-means algorithm is affected by the initial clustering center during segmentation, and its segmentation result is not ideal. In addition, the algorithm ignores the position information of the image, which leads to a high segmentation error [31]. Compared with the mean shift algorithm, the k-means algorithm based on custom initial clustering centers proposed in this research had a better effect on image segmentation. When performing initial segmentation of the image, this improved k-means algorithm makes full use of the distribution information of the data set and selects the data object with relatively large local density as the initial clustering center, thereby optimizing the algorithm and reducing the possibility of dividing the image by mistake. This method of finding the initial cluster centers is more efficient than the random method, and it is not easy to fall into a local minimum, making this experiment more stable [32, 33].

## 5. Conclusion

This research explored the effect of regular dialysis on the cranial nerves of patients with ESRD based on rs-fMRI and central k-means algorithm. It was found that this improved k-means algorithm showed better time efficiency and lower error rate when rs-fMRI was adopted to diagnose the effect of regular HD on the brain function of ESRD patients. Compared with normal volunteers, ESRD patients had poor neuropsychological cognitive function. The rs-fMRI scan of the brain showed that the abnormal brain area of the experimental group mainly appeared in the default network area of the brain, namely, the medial prefrontal lobe and the anterior cuneiform lobe/posterior cingulate. This means that the abnormality of FC in a certain part of the brain can detect the neuropathological basis of early cognitive dysfunction in patients. Due to the small number of samples in this research, the samples and results showed low overall representativeness. The inclusion criteria for ESRD patients ignored the effects of antihypertensive and hypoglycemic drugs taken by the patients on brain function, and the indicators for neuropsychological cognitive assessment of the two groups of patients were also relatively limited. In the follow-up research, it would be necessary to increase the blood biochemistry index for detecting normal volunteers and analyze its correlation with the results of neuropsychological cognitive assessment. In conclusion, this research provided data support for the clinical rs-fMRI diagnosis of the effect of regular HD on the brain function of ESRD patients and the mechanism of the occurrence of cognitive dysfunction in patients.

## Figures and Tables

**Figure 1:** The clustering process of initial k-means algorithm.

**Figure 2:** MRI scan of a patient's brain. (a) was a normal MR scan; (b) was an MRI scan after k-means clustering.

**Figure 3:** The operation flow chart of the improved k-means algorithm for custom clustering centers.

**Figure 4:** Comparison on running time between the improved and traditional k-means algorithms. 1 and 2 referred to the images with size of 256 × 256, 3 and 4 referred to the image in 512 × 512). ∗Compared with traditional k-means algorithms, *P* < 0.05.

**Figure 5:** Comparison on segmentation error rate among three different algorithms. ∗Compared with other algorithms, *P* < 0.05.

**Figure 6:** Comparison on age, years of education, height, and weight of the two groups of subjects.

**Figure 7:** Test results of DSST scale and MoCA scale. ∗Compared with the control group, *P* < 0.05.

**Figure 8:** Correlation between the blood biochemistry results and the DSST scale and MoCA scale.

**Figure 9:** Analysis on the results of the functional connectivity difference between two groups. (a) showed the functional connectivity difference; (b) showed the X, Y, and Z axis of the MNI. ∗Compared with the control group, *P* < 0.05.

## Data Availability

The data used to support the findings of this study are available from the corresponding author upon request.
